# Analysis of the Prognostic Impact of Staged Nursing Interventions on the Treatment of Patients with COPD Combined with Type II Respiratory Failure

**DOI:** 10.1155/2022/4498161

**Published:** 2022-07-19

**Authors:** Yun Zheng, Haihua Wu

**Affiliations:** ^1^Pulmonary and Critical Care Medicine, TongDe Hospital, Zhejiang Province, China; ^2^Emergency Department, Tongde Hospital, Zhejiang Province, China

## Abstract

**Objective:**

To analyze the prognostic impact of staged nursing interventions on the treatment of patients with chronic obstructive pulmonary diseases (COPD) combined with type II respiratory failure.

**Methods:**

120 patients with COPD combined with type II respiratory failure admitted to our hospital between January 2021 and January 2022 were divided into a control group and a study group, with 60 patients in each group. The control group received conventional strategy interventions, and the study group received staged nursing interventions. Pulmonary function, blood gases, health impairment, knowledge, mood, hope level, and quality of survival were evaluated before and after patient care, and satisfaction and the impact on patient prognosis were assessed.

**Results:**

The improvement of pulmonary function and blood gas in the study group was better than that in the control group aftercare, and the difference was statistically significant (*P* < 0.05). Health impairment and mood scores were lower in the study group compared to the control group aftercare, and the difference was statistically significant (*P* < 0.05). Knowledge awareness, hope, and quality of survival scores were higher in the study group compared to the control group aftercare, with statistically significant differences (*P* < 0.05). The rate of excellent prognosis and satisfaction was higher in the study group compared with the control group, and the difference was statistically significant (*P* < 0.05).

**Conclusion:**

The implementation of staged nursing interventions during the treatment of patients with COPD combined with type II respiratory failure can significantly improve patient prognosis and has a high application value.

## 1. Introduction

Chronic obstructive pulmonary disease (COPD) is a chronic respiratory disease with high mortality and recurrence rates, which is characterized by decreased lung function and incomplete reversible airflow obstruction. Studies have concluded [1] that the aggravation of airway obstruction in patients affects the ventilation function and eventually leads to the development of type II respiratory failure, which has a certain impact on the life safety of patients. Currently, the treatment of COPD combined with type II respiratory failure is mainly based on noninvasive ventilation therapy, which can not only effectively relieve airway obstruction but also inhibit further aggravation of respiratory failure, with significant clinical efficacy [2]. However, it has been reported [3] that in order to effectively improve the efficacy of mechanical ventilation therapy in patients, reasonable and effective nursing interventions are needed to maximize the effect of ventilation and improve the prognosis.

The main contents of staged nursing intervention include admission education and management, operation period nursing, early postoperative rehabilitation nursing, and continuous rehabilitation nursing guidance. According to different surgical approaches and repair methods, targeted care, especially postoperative rehabilitation care and functional exercise, can greatly promote the recovery of patients' functions and shorten the patient's hospital stay. In contrast, routine care mainly reffered to admission guidance, simple health education, regular physical examination, prevention of complications, and guidance of patients on the use of COPD medication, which was demonstrated to be less efficient than staged nursing intervention [4]. As shown in a study of nursing intervention on self-efficacy among elderly patients with acute coronary syndrome after percutaneous coronary intervention, the nursing intervention effect of the 2 groups after intervention was improved before intervention (*P* < 0.05), and the hospital anxiety and depression scale (HADS) was lower than that of the control group after psychological intervention. The general self-efficacy scale scores of experimental group were obviously improved after receiving the intervention, and the scores in the experimental group were much higher than the control group after receiving the intervention, namely *P* < 0.05 [1]. Inspired by these data of the prognostic effect of nursing interventions, this study is aimed at investigating the effectiveness of its application by adding staged nursing interventions during patient treatment, which is reported as below.

## 2. Objects and Methods

### 2.1. Object of the Study

120 patients with COPD combined with type II respiratory failure who met the inclusion and exclusion criteria and were admitted to our hospital between January 2021 and January 2022 were selected and divided into a control group and a study group of 60 cases each according to the random number table method. The general information of the two groups is shown in Table 1, and the two groups were balanced and comparable (*P* > 0.05). The inclusion criteria are as follows: meeting the clinical diagnostic criteria for COPD and type II respiratory failure, complete information, voluntary participation, and all treated with the same treatment protocol. The exclusion criteria are as follows: having other pulmonary pathologies such as pulmonary embolism; lung cancer; aberrant cardiogenic pulmonary edema; liver, kidney, and another important organ insufficiency; blurred consciousness; and no communication ability.

### 2.2. Methods

#### 2.2.1. Treatment Method

Both groups were treated with conventional interventions, including nutritional support and water-electrolyte balance, and were treated with a dual-level noninvasive ventilator, with 12 breaths/min to 20 breaths/min, 6 cm H_2_O to 8 cm H_2_O as the initial inspiratory pressure, and 2 cm H_2_O to 3 cm H_2_O as the initial inspiratory pressure, and the patients were closely monitored for changes in their condition during treatment, and the parameters were adjusted in time. The maximum inspiratory air pressure was 5 cm H_2_O~6 cm H_2_O, and when the patient's condition was in a stable state, the inspiratory air pressure and suction pressure were adjusted down, and the inspiratory oxygen level was 40% during this process, and the flow rate was 4 L/min~6 L/min, and ventilation was performed for 4 h ~6 h each time.

#### 2.2.2. Nursing Method

In the control group, the general routine strategy interventions such as disease monitoring and complication prevention were performed, disease monitoring was done according to medical prescriptions, and patients were closely monitored for the presence of sputum in the respiratory tract and cleared in time to reduce the occurrence of adverse events.

The study group applied the stage nursing strategy intervention and formed a stage nursing team, which consisted of a department physician, a department nurse manager, and 5 nurses with more than 5 years of experience in respiratory medicine and excellent service attitude. The nurse manager, as the team leader, discussed the nursing interventions with the team members and formulated the stage nursing measures, which were specifically implemented by the nurses. The specific measures are shown in Table 2.

### 2.3. Indicator Observation

#### 2.3.1. Pulmonary Function, Blood Gas Analysis

Pulmonary function and arterial blood gas stability were measured using a pulmonary function and fully automated blood gas analyzer (GEM Premier 4000) before the patients were admitted to the group (before care) and before they were discharged from the hospital (aftercare). Pulmonary function was evaluated based on FEV1, FVC, and FEV1/FVC, and arterial blood gas stability was evaluated based on PaO_2_, SaO_2_, and PaCO_2_ levels.

#### 2.3.2. St. George's Respiratory Questionnaire (SGRQ) Evaluation

The health impairment of patients before and after patient care was evaluated based on the St. George's Respiratory Questionnaire (SGRQ) [5], which includes dimensions such as disease impact on life, activity limitation, and respiratory condition. The entire scale consists of 50 questions, where the lowest and highest scores on the scale are 0 and 100, respectively, with lower scores indicating less health damage to the patient from the disease.

#### 2.3.3. Evaluation of Knowledge of Pulmonary Rehabilitation

Before and after the patients' care, the patients' knowledge was evaluated based on the scores of our self-made pulmonary rehabilitation knowledge questionnaire, which consisted of 5 items: diet, medication, disease, exercise, and oxygen therapy. The entire scale consisted of 24 questions, where the lowest and highest scores of the scale were 0 and 24, respectively, with lower scores indicating more desirable patient perceptions of the disease.

#### 2.3.4. Emotion, Hope Level Evaluation

The patient's mood and hope level were evaluated before and after patient care using the Self-Rating Scale for Depression (SDS), Self-Assessment Scale for Anxiety (SAS), and Herth Hope Scale developed by Zung, respectively; SDS and SAS both contain 20 questions and are rated on a 4-point scale, with lower scores indicating weaker depression and anxiety. The Herth Hope Scale consists of 12 questions, with scores of 12-23 being low, 24-35 being moderate, and 36-48 being high, with higher scores indicating a higher level of hope.

#### 2.3.5. Survival Quality Evaluation

The quality of survival was evaluated on the Quality of Survival Scale before and after patient care, with a total of 26 questions on a 5-point scale, with each question scoring 0-5, with higher scores indicating better quality of survival.

#### 2.3.6. Prognostic Evaluation

The occurrence of adverse events such as multiple organ failure, cardiovascular disease, and death that occurred before the patient was admitted to the hospital for treatment until discharge was used as a prognostic evaluation criterion, and the occurrence was considered a poor prognosis, and the opposite was considered an excellent prognosis.

#### 2.3.7. Nursing Satisfaction Evaluation

Patients in both groups were assessed for nursing satisfaction by our questionnaire, which included 4 items, namely, very satisfied, satisfied, dissatisfied, and very dissatisfied, and (very satisfied + satisfied)/the total number of cases ×100% = total satisfaction.

### 2.4. Statistical Analysis

SPSS22.0 statistical software was used for analysis and processing. The Kolmogorov-Smirnov test was applied to test whether the data conformed to a normal distribution, and the measurement data conforming to normal distribution were described by the mean ± standard deviation ($\bar{x}\pm s$), and the independent samples *t*-test was used for comparison between groups, and the paired *t*-test was used for comparison before and after patient care; median and quartile spacing M (Q1, Q3) were applied for those not conforming to the normal distribution, and Wilcoxon's comparison was used between groups. Count data were expressed as *n* (%), *χ*^2^ test. *P* < 0.05 was considered statistically significant.

## 3. Results

### 3.1. Comparison of Pulmonary Function Indexes between the Two Groups

The comparison of pulmonary function between the two groups before care was not significant (*P* > 0.05); after care, the pulmonary function of the two groups was higher than before care, and the increase was more significant in the study group compared with the control group (*P* < 0.05). See Table 3 and Figure 1.

### 3.2. Comparison of Blood Gas Indicators between the Two Groups

The comparison of blood gases between the two groups before care was not significant (*P* > 0.05); after care, the blood gas indexes of the two groups were higher than before care, and the increase was more significant in the study group compared with the control group (*P* < 0.05). See Table 4 and Figure 2.

### 3.3. Comparison of SGRQ Scores for Health Impairment between the Two Groups

The comparison of SGRQ scores of health impairment between the two groups before care was not significant (*P* > 0.05); after care, the SGRQ scores of health impairment in both groups were lower than before care, and the reduction was more significant in the study group compared with the control group (*P* < 0.05). See Table 5 and Figure 3.

### 3.4. Comparison of Knowledge Awareness Scores of Pulmonary Rehabilitation between Two Groups

The comparison of the knowledge scores of the two groups before care was not significant (*P* > 0.05); after care, the knowledge scores of the two groups were higher than before care, and the increase was more significant in the study group compared with the control group (*P* < 0.05). See Table 6 and Figure 4.

### 3.5. Comparison of Mood and Hope Scores between the Two Groups

The comparison of mood and hope scores between the two groups before care was not significant (*P* > 0.05); after care, the hope scores of the two groups were higher than before care, and the increase was more significant in the study group compared with the control group (*P* < 0.05); after care, the mood scores of the two groups were lower than before care, and the decrease was more significant in the study group compared with the control group (*P* < 0.05). See Table 7 and Figure 5.

### 3.6. Comparison of the Quality of Survival between the Two Groups

The comparison of the quality of survival scores between the two groups before care was not significant (*P* > 0.05); after care, the quality of survival in both groups was higher than before care, and the increase was more significant in the study group compared with the control group (*P* < 0.05).  Table 8, Figure 6.

### 3.7. Comparison of Prognosis between the Two Groups

The study group had a higher rate of excellent prognosis than the control group (*P* < 0.05). See Table 9.

### 3.8. Comparison of Nursing Satisfaction between the Two Groups

Nursing satisfaction was higher in the study group than in the control group (*P* < 0.05). See Table 10.

## 4. Discussion

Currently, the treatment of patients with COPD combined with type II respiratory failure is based on noninvasive ventilation, which is the most commonly used treatment for this disease, and this method has the advantages of easy operation, ready access to the machine, and low trauma to the patient's organism, which can continuously improve the patient's hypoxia and respiratory function after application [1, 4, 5]. However, studies have shown [6] that some patients have varying degrees of psychological negativity in the early stages of treatment, which affects the effect of ventilation and increases the risk of poor prognosis, so appropriate nursing interventions need to be given to patients during treatment to improve the prognosis.

Most of the conventional nursing tools currently used in the clinic are based on the patient's condition in order to maintain treatment, ignoring to some extent the differences in patients' stage needs [7–9]. Stage-based nursing measures are the hotspot studied at present, which was reported [10] that such nursing means can implement targeted measures and interventions at different stages. Duiring the nursing process, the psychological and physiological characteristics of patients are fully considered, which aimed to obtain the rapid disease recovery from early to late stages. Unlike conventional nursing measures, the stage nursing measures have clearer goals and are related to the patient's disease recovery process, and are progressive nursing measures with ideal clinical application value [11, 12]. In this paper, the study group performed targeted noninvasive ventilation care in the early, middle, and late stages of treatment to avoid disease deterioration during the stabilization phase and to focus on postwithdrawal respiratory function training during the late withdrawal process. The improvement in pulmonary function and blood gases was found to be more significant in the study group than in the control group aftercare, a result that may be related to the fact that the study group was more effective in diagnosing the patient's specific disease at multiple stages of care.

It has been reported [13] that some patients develop psychological negativity and lose their level of hope after the onset of the disease due to the fear of not recovering from the disease. The results of this study showed that patients who applied staged care had significantly reduced negative psychological emotions and increased their hope levels, suggesting that staged care may increase hope levels and alleviate negative psychological emotions by promoting patients' recovery from disease. In addition, the clinical evaluation of the effectiveness of treatment is mostly based on the prognosis of the patients [14]. Therefore, this study further analyzed the impact of patient stage care measures on patient prognosis, which showed that patients in the study group had a higher rate of excellent prognosis. This result is consistent with the fact that care measures can improve the prognosis in both physiological and psychological aspects.

In conclusion, staged nursing interventions can significantly improve pulmonary function and blood gases and improve treatment prognosis in patients with COPD combined with type II respiratory failure with ideal results.

## Figures and Tables

**Figure 1:** Histogram comparing pulmonary function before and after patient care in the two groups.

**Figure 2:** Histogram of blood gas comparison between two groups before and after patient care.

**Figure 3:** Histogram comparing SGRQ scores of health impairment in the two groups.

**Figure 4:** Histogram comparing the knowledge scores of pulmonary rehabilitation between the two groups.

**Figure 5:** Histogram comparing the mood and hope scores of the two groups.

**Figure 6:** Histogram comparing the quality of survival scores before and after patient care for the two groups.

**Table 1:** Comparison of general information between the two groups [$\bar{x}\pm s$_,_*n*(%)].

General information	Control group (*n* = 60)	Study group (*n* = 60)	*χ* ^2^/t	*P*
Gender				
Male	24(40.00)	28(46.67)	0.543	0.461
Female	36(60.00)	32(53.33)		
Average age (years)	58.06 ± 4.56	58.11 ± 4.32	0.062	0.951
Average BMI (kg/m^2^)	23.54 ± 2.31	23.67 ± 2.43	0.300	0.764
Duration of COPD (years)	5.12 ± 0.78	5.17 ± 0.80	0.347	0.729
Duration of respiratory failure (d)	8.93 ± 1.12	9.11 ± 1.16	0.865	0.389
Degree of dyspnea				
Moderate	45(75.00)	41(68.33)	0.657	0.418
Severe	15(25.00)	19(31.67)		
Educational level				
Junior high school and below	17(28.33)	16(26.67)	0.962	0.618
Secondary and high school	21(35.00)	26(43.33)		
College and above	22(36.67)	18(30.00)		
Combined diabetes	6(10.00)	7(11.67)	0.086	0.769
Combined hypertension	8(13.33)	7(11.67)	0.076	0.783
Combined hyperlipidemia	10(16.67)	9(15.00)	0.062	0.802
APACHE II score (points)	20.71 ± 2.31	20.89 ± 2.34	0.424	0.672

**Table 2:** Specific care measures.

Implementation phase	Measures
Initial stage	At the initial stage of noninvasive ventilation, the nurse should give the patient a brief education about the necessity and safety of noninvasive ventilation to avoid emotional fluctuations. The mask should be selected according to the patient's face shape to avoid mask leakage, the appropriate tightness should be adjusted, and the sponge or gauze should be placed on the patient's frontal bone and nasal bridge.

Medium stage	This stage is 2 h after the patient's noninvasive ventilation until the disease is stable. At this time, observe the patient's adaptation to noninvasive ventilation, in order to avoid the patient's agitation, divert the patient's attention during this process, and elevate the head of the bed according to the patient's acceptance, and keep the patient's head and neck and airway vertical. Pay attention to whether there is sputum in the patient's airway, and if there is sputum, remove it in time to avoid the airway being obstructed.

Late stage	This stage is from the patient's disease stabilization to the ventilator withdrawal stage. (i) Withdrawal care: before withdrawing the ventilator, comprehensively assess whether the patient meets the withdrawal criteria, explain to the patient in detail the reasons and precautions for withdrawal, monitor the vital signs in real-time during the withdrawal process, and be prepared to get on the ventilator again at any time. (ii) Psychological guidance: pay close attention to the psychological and emotional changes of the patients, use visual simulation scoring to rate the patients' psychological state, and grade the care according to the score. <2 points for level 1 psychological care, use common psychological care, focus on the establishment of a sense of security when caring for the patients, focus on the current problems that the patients have, and understand the underlying causes of the patients' psychological problems. Use comfort, communication, and explanation to give patients psychological support and improve their sense of security. 2 points ≤ score < 4 points for level 2 psychological care, use mental relaxation method to improve patients' psychology and use light music in a quiet environment to allow patients to achieve a state of general relaxation to relieve mental tension and improve psychology. ≥4 points of level 3 psychological care to give patients family support, build confidence, and relieve negative emotions. During the implementation process, patients were made aware of the adverse psychological effects on recovery after treatment to establish a correct positive mindset.

Later consolidation care	In the later stage, we did the consolidation nursing intervention of respiratory function exercise, recorded the patient's respiratory function exercise daily, actively guided and helped the patient in the process of exercise, did about 0.5 h of exercise each time, and performed 3-5 times of exercise daily. During the exercise process, patients were encouraged appropriately according to their positive degree of exercise, so as to improve their compliance with exercise and promote rapid recovery from disease.

**Table 3:** Comparison of lung function between the two groups ($\bar{x}\pm s$).

Group	FEV_1_(L)		FVC(L)		FEV_1_/FVC(%)	
	Before nursing	After nursing	Before nursing	After nursing	Before nursing	After nursing
Control group (*n* = 60)	1.32 ± 0.24	1.72 ± 0.25	1.97 ± 0.22	2.32 ± 0.25	66.14 ± 5.62	72.61 ± 4.91
Study group (*n* = 60)	1.33 ± 0.21	2.46 ± 0.16	1.99 ± 0.19	2.85 ± 0.31	66.21 ± 5.49	76.84 ± 5.04
*t*	0.243	19.310	0.533	10.310	0.069	4.657
*P*	0.809	0.001	0.595	0.001	0.945	0.001

**Table 4:** Comparison of blood gas indicators between the two groups ($\bar{x}\pm s$).

Group	PaCO_2_ (mmHg)		PaO_2_ (mmHg)		SaO_2_ (%)		PH	
	Before nursing	After nursing	Before nursing	After nursing	Before nursing	After nursing	Before nursing	After nursing
Control group (*n* = 60)	72.38 ± 7.26	62.82 ± 6.04	52.62 ± 5.49	67.03 ± 6.56	74.39 ± 4.85	82.31 ± 4.91	7.18 ± 0.05	7.34 ± 0.03
Study group (*n* = 60)	73.09 ± 7.14	51.96 ± 4.31	52.93 ± 5.52	81.14 ± 7.06	73.76 ± 4.32	94.82 ± 4.71	7.19 ± 0.04	7.48 ± 0.06
*t*	0.540	11.340	0.308	11.340	0.747	14.240	1.210	16.170
*P*	0.590	0.001	0.758	0.001	0.457	0.001	0.229	0.001

**Table 5:** Comparison of SGRQ scores for health impairment between the two groups [($\bar{x}\pm s$), points].

Group	Breathing conditions		Restricted activities		Disease impact on life		Total score	
	Before nursing	After nursing	Before nursing	After nursing	Before nursing	After nursing	Before nursing	After nursing
Control group (*n* = 60)	64.82 ± 7.45	48.39 ± 6.98	69.31 ± 8.14	57.08 ± 7.43	61.41 ± 8.04	49.32 ± 6.53	67.09 ± 9.15	54.51 ± 7.11
Study group (*n* = 60)	65.12 ± 8.07	44.52 ± 6.21	71.12 ± 8.21	51.42 ± 7.22	61.52 ± 8.11	43.15 ± 6.41	66.35 ± 9.26	46.41 ± 6.26
*t*	0.212	3.209	1.213	4.232	0.075	5.223	0.440	6.623
*P*	0.833	0.002	0.228	0.001	0.941	0.001	0.661	0.001

**Table 6:** Comparison of pulmonary rehabilitation knowledge scores between the two groups [($\bar{x}\pm s$), points].

Group	Diet knowledge		Medication knowledge		Disease knowledge		Sports knowledge		Oxygen therapy knowledge		Total score	
	Before nursing	After nursing	Before nursing	After nursing	Before nursing	After nursing	Before nursing	After nursing	Before nursing	After nursing	Before nursing	After nursing
Control group (*n* = 60)	1.31 ± 0.65	2.05 ± 0.71	2.01 ± 1.04	2.73 ± 1.11	4.19 ± 1.55	5.03 ± 1.59	2.39 ± 1.12	3.14 ± 1.08	1.24 ± 0.48	1.91 ± 0.42	11.14 ± 1.36	14.86 ± 2.57
Study group (*n* = 60)	1.29 ± 0.67	2.39 ± 0.66	2.04 ± 1.02	3.65 ± 1.07	4.16 ± 1.54	6.71 ± 1.46	2.41 ± 1.07	4.11 ± 1.28	1.22 ± 0.46	2.52 ± 0.42	11.12 ± 1.42	19.35 ± 2.96
*t*	0.166	2.717	0.160	4.622	0.106	6.028	0.100	4.486	0.075	7.955	0.079	8.872
*P*	0.868	0.008	0.874	0.001	0.915	0.001	0.921	0.001	0.941	0.001	0.937	0.001

**Table 7:** Comparison of emotions and hopes between the two groups [($\bar{x}\pm s$), points].

Group	Hopes								SAS		SDS	
	Attitude towards reality and the future		Adopt an affirmative action attitude		The attitude of maintaining a close relationship with others		Total score					
	Before nursing	After nursing	Before nursing	After nursing	Before nursing	After nursing	Before nursing	After nursing	Before nursing	After nursing	Before nursing	After nursing
Control group (*n* = 60)	10.21 ± 1.96	11.95 ± 1.14	10.24 ± 1.52	12.24 ± 1.05	12.17 ± 0.53	13.38 ± 1.05	33.42 ± 3.62	37.49 ± 3.28	50.13 ± 6.81	39.62 ± 4.62	44.35 ± 6.45	40.43 ± 4.05
Study group (*n* = 60)	10.29 ± 1.82	14.27 ± 1.22	10.31 ± 1.23	14.39 ± 1.19	12.15 ± 0.62	15.31 ± 1.56	33.35 ± 3.12	45.03 ± 4.41	50.64 ± 6.37	35.79 ± 4.14	45.34 ± 6.17	35.71 ± 3.73
*t*	0.232	10.760	0.277	10.490	0.190	7.950	0.114	10.630	0.424	4.782	0.859	6.640
*P*	0.817	0.001	0.782	0.001	0.850	0.001	0.910	0.001	0.673	0.001	0.392	0.001

**Table 8:** Comparison of quality of survival scores before and after patient care between the two groups [($\bar{x}\pm s$), points].

Group	Physiological field		Psychological field		Social field		Circumstance field		Total score	
	Before nursing	After nursing	Before nursing	After nursing	Before nursing	After nursing	Before nursing	After nursing	Before nursing	After nursing
Control group (*n* = 60)	9.29 ± 1.03	11.32 ± 1.57	9.18 ± 1.05	12.57 ± 2.18	10.33 ± 1.53	13.52 ± 2.16	11.38 ± 1.08	13.24 ± 1.87	38.79 ± 5.13	48.67 ± 4.37
Study group (*n* = 60)	9.25 ± 1.12	14.68 ± 2.54	9.12 ± 1.03	15.68 ± 2.34	10.24 ± 1.12	16.16 ± 2.48	11.34 ± 1.12	15.63 ± 3.24	38.62 ± 5.22	62.57 ± 8.49
*t*	0.204	8.716	0.316	7.533	0.368	6.218	0.199	4.949	0.180	11.280
*P*	0.839	0.001	0.753	0.001	0.714	0.001	0.842	0.001	0.958	0.001

**Table 9:** Comparison of prognosis between the two groups (n, %).

Group	Poor prognosis	Good prognosis
Control group (*n* = 60)	11(18.33)	49(81.67)
Study group (*n* = 60)	3(5.00)	57(95.00)
*χ* ^2^	5.175	
*P*	0.023	

**Table 10:** Comparison of nursing satisfaction between the two groups (n, %).

Group	Very satisfied	Satisfied	Dissatisfied	Very dissatisfied	Nursing satisfaction (%)
Control group (*n* = 60)	35	13	7	5	48(80.00)
Study group (*n* = 60)	40	17	2	1	57(95.00)
*χ* ^2^					6.171
*P*					0.013

## Data Availability

The data used to support this study is available from the corresponding author upon request.
